# Evaluation of MWCNT Particles-Reinforced Magnesium Composite for Mechanical and Catalytic Applications

This article has been retracted.

**DOI:** 10.1155/2022/7773185

**Published:** 2022-05-24

**Authors:** T. Sathish, Vinayagam Mohanavel, Palanivel Velmurugan, Saleh Alfarraj, Sami Al Obaid, Shanmugam Sureshkumar, J. Isaac Joshua Ramesh Lalvani

**Affiliations:** ^1^Department of Mechanical Engineering, Saveetha School of Engineering, SIMATS, Chennai 602105, Tamil Nadu, India; ^2^Centre for Materials Engineering and Regenerative Medicine, Bharath Institute of Higher Education and Research, Chennai 600073, Tamil Nadu, India; ^3^Department of Mechanical Engineering, Chandigarh University, Mohali 140413, Punjab, India; ^4^Zoology Department, College of Science, King Saud University, Riyadh 11451, Saudi Arabia; ^5^Department of Botany and Microbiology, College of Science, King Saud University, PO Box -2455, Riyadh -11451, Saudi Arabia; ^6^Department of Animal Resources Science, Dankook University, 119 Dandae-ro, Cheonan 31116, Republic of Korea; ^7^Department of Mechanical Engineering, Faculty of Mechanical and Production Engineering, AMIT, Arbaminch University, Arba Minch, Ethiopia

## Abstract

Aluminum, magnesium, and copper materials must have increased mechanical strength with enhanced wear and corrosion resistance. Substantial research focused on reinforcing hard particles into low-strength materials using stir casting or powder metallurgy. This work is intended to develop the magnesium hybrid matrix with the dispersion of boron carbide (B_4_C) and multiwall carbon nanotubes (MWCNTs). Hybrid magnesium composites are prepared, although the powder metallurgy route considers different process parameters. Statistical analysis such as Taguchi L16 orthogonal array is involved in this work. It is used to find the magnesium hybrid samples' minimum and maximum wear, corrosion, and microhardness levels. Powder metallurgy parameters are B_4_C (3%, 6%, 9%, and 12%), MWCNT (0.2%, 0.4%, 0.6%, and 0.8%), ball milling (1, 2, 3, and 4 h), and sintering (3, 4, 5, and 6 h). The ball milling parameters are extremely influenced in the wear test analysis. Minimum wear losses are obtained as 0.008 g by influencing the 4 h ball milling process. Similarly, 3 h of sintering time offered a minimum corrosion rate of 0.00078 mm/yr. In microhardness analysis, the percentage of MWCNTs is highly implicated in narrow hardness resulting in the hardness value of 181. The hardness value is recorded using 0.2% MWCNTs in the magnesium alloy AZ80.

## 1. Introduction

Compared to pure metals or alloys, metal-matrix composites have excellent advantages due to their mechanical properties such as corrosion, wear, creep, and hardness [1]. Aluminum alloys are widely used in the industry and automotive sectors. The strength of aluminum is increased through reinforced particles, namely, boron carbide, silicon carbide, zirconium oxide, aluminum oxide, etc. [2–4]. Since they are expensive, these reinforcement particles are to be replaced with fly ash and natural minerals. In India, fly ash is obtained from the thermal power plant in a massive amount. Modern trends need more lightweight materials to make numerous parts for householding applications, vehicle construction, and aerospace applications [5]. Compared to aluminum material, magnesium has low weight and low density (1.738 g/cm); like the way, the magnesium possesses a considerable property than aluminium that is biocompatible [6]. Strengthening magnesium alloy by using various reinforcing ceramic particles, carbon fibers, etc. is also performed [7]. Novel research is undertaken to improve the strength of the magnesium alloy by adding graphene nanoparticles and carbon nanotubes [8–10]. The CNTs are the most wanted nanoparticles among all reinforced particles due to their excellent large surface area and superior mechanical, electrical, thermal, and optical properties [11]. The CNT has excellent ultrahigh strength, and it is served in electrical and electronics applications such as sensors, voltage inverters, and transistors [12–14]. Many researchers conducted experimental work based on the CNT's reinforcement. The different melting processes are concentrated to melt the CNTs and obtain uniform dispersion in the matrix material [15]. In the powder metallurgy process, the CNT support to the matrix material has offered excellent hybrid composite materials [16]. In current years, magnesium alloy is consumed chiefly due to its lightweight, extreme strength, and biodegradable nature. The addition of reinforced particles into the magnesium alloy improves the properties of the magnesium alloy. Carbon nanotubes (CNTs) have excellent material qualities, such as low density, extreme tensile strength, and excellent thermal conductivity. Hence, it is used to make metal-matrix composites (MMCs). In the magnesium alloy, a tiny amount of CNT reinforcement can enhance the mechanical and physical properties. Most research studies use ceramic particles and CNTs as reinforced particles. From an extensive literature study, the research gap is identified that a few of the results only considered MWCNTs. Hence, this work focused on ring high-strength magnesium alloy composites by adding boron carbide with MWCNT through the P/M route. AZ80 magnesium alloy possesses incorporated mechanical properties: high strength, excellent plasticity, and toughness. Hence, this research work considered the AZ80 matrix phase alloy, which is used in the fabrication of biomedical instruments. Increasing wear and corrosion resistance of AZ80 for medical applications is achieved by reinforcement with boron carbide and MWCNT. This work is significant for the fabrication of bone repairing plates and bone screws and biomedical applications; hence, this work was undertaken to focus on the novelty of preparation for hybrid composites. The wonder of this investigation is the addition of ceramic materials such as boron carbide and multiwall carbon nanotubes (MWCNTs) into the AZ80 to obtain excellent properties.

This work aims to fabricate magnesium matrix composites by adding different percentage levels of boron carbide and MWCNTs. The powder metallurgy process is involved in this work to make excellent magnesium composites with Taguchi optimization. Furthermore, the wear, corrosion, and microhardness tests were conducted on the prepared magnesium composites.

## 2. Materials and Methods

Magnesium alloy AZ80 is selected for this experimental work; it is silvery-white and contains aluminum, zinc, manganese, copper, silicon, iron, and nickel. AZ80 is lightweight and has good machinability characteristics; it is produced by sintering technology [17–19]. Typically, magnesium alloy is lightweight in nature; nanoparticles should be added to it to improve its properties. Nanoparticle additions improve the properties of the magnesium alloy, such as tensile hardness, wear, and corrosion. Magnesium alloy AZ80 is procured from the Jagada Industries, Virudhunagar, and boron carbide powder 2 kg is purchased from Ceramics International, Salem. Hydra-reinforced nanomaterials such as multiwall carbon nanotubes (MWCNTs) strengthened magnesium composites. The MWCNTs are purchased from Fiber Region, Valasarvakkam, Chennai. MWCNTs are multiwalled, with purity >98 percentage carbon basis, O.D. × L of 6−13 nm × 2.5–20 *μ*m, respectively [20–22]. The powder metallurgy process is used to prepare the magnesium hybrid composites with the assistance of the ball milling process. Mixed powders are compacted well; the green compacting specimens are sintered with the influence of argon gas.  Table 1 presents the composition of AZ80 magnesium alloy.

Table 2 presents the process parameters of the powder metallurgy process by applying four parameters and four levels, such as L16 OA [23–25].

## 3. Experimental Procedure

The magnesium hybrid composites are made from AZ80 magnesium alloy with the addition of 3%, 6%, 9%, and 12% of boron carbide (9.25 (0.2%, 0.4%. 0.6%, and 0.8%) diameter) and multiwall carbon nanotubes (0.2%, 0.4%. 0.6%, and 0.8%) [26–28]. Nanotubes' specifications are 10–15 nm of outer diameter, 3–8 nm of inner diameter, and 0.1–12 *µ*m in length. The powders are mixed well under inhomogeneous conditions using a planetary ball mill, as shown in Figure 1. The ball milling speed is fixed at 300 pm, and the steel balls of 5 mm and 10 mm are placed inside the mill for homogeneous mixing [29–31]. The ball milling process is conducted for 1, 2, 3, and 4 h. Additionally, 5% of methanol is added to avoid the agglomeration of the powder. After milling, the powders are compacted through a cold compaction process by applying a 300 MPa load to prepare the green compact, as shown in Figure 2.

Furthermore, the sintering process is carried out to convert the compact green specimen into a helpful test specimen [32–34]. The samples are sintered for different time periods such as 3, 4, 5, and 6 h maintaining 4°C. Argon gas is supplied to the furnace during the sintering process.  Figure 3 presents the sintering furnace, and Figure 4 illustrates the before and after sintering specimens [35–37].

The tribological experiment is conducted through the DUCOM model dry sliding pin on the disc wear test apparatus, as shown in Figure 5. Wear test specimens are prepared from the extruded samples per the ASTM G99. The dimensions of the specimens are 12 mm in diameter and 35 mm in length [38, 39]. Parameters of the wear test are a load of 30 N, sliding velocity of 2 m/s, and sliding distance of 1200 m. Using a digital weighing balance, the before and after weight of the specimens were determined for evaluating the mass loss and wear [40–42].

The microhardness test is conducted using a Vickers hardness tester for the Digital Micro Vickers Hardness Tester model. The specifications of the Vickers hardness tester are voltage 220 V, power 1500 W, and frequency 60 Hz. All the samples are tested three to four times, and the hardness value is averaged [43]. A salt spray corrosion test is conducted with the help of the Weiss model salt spray chamber; the frequency range is 50/60 Hz. All the samples are hung inside the groomer with a continuous circulation of 5% of NaCl solution by using the pump, and the time is maintained as 72 hours [44]. After 24 h, the samples were taken from the chamber and cleaned thoroughly for further weight measurement; the mass loss was measured with the help of a 0.01 g-resolution digital balance for estimating the corrosion rate [45].

## 4. Results and Discussion

The results of the wear test and the microhardness and corrosion rates are presented in Table 3. The minimum wear was 0.007 g with the influence of 9% boron carbide, 0.8% MWCNT, 2 h of the ball milling process, and 3 h of the sintering process. The maximum wear was 0.0047 g. In the microhardness analysis, the maximum hardness was 181.4 HV by 12% of boron carbide, 0.2% of MWCNT, 4 h of the ball milling process, and 4 h of the sintering process. On the other hand, the minimum microhardness was recorded at 84.3 HV. The minimum corrosion rate was registered at 0.00078 mm/yr from the corrosion rate examination by 12% boron carbide, 0.4% of MWCNT, 3 h of the ball milling process, and 3 h of the sintering process. The maximum corrosion rate was recorded at 0.00827 mm/yr.

### 4.1. Wear Analysis

In wear analysis, the ball milling parameter has a significant influence. It was considered the priority paramter among the four parameters. The influencing order of the parameters is illustrated in Table 4 (mean) and Table 5 (S/N ratio).

Furthermore, the ranks of the parameters were concluded as follows: the MWCNT percentage was ranked second, the sintering time parameter was ranked third, and the boron carbide percentage was ranked fourth. Minimum wear was attained by the influencing optimal parameters such as 6% boron carbide, 0.8% MWCNT, 1 h of on the ball milling process, and 3 h of the sintering process. The influence of MWCNT % was ranked as the second parameter in the wear analysis; in general, the MWCNT possesses high strength compared to B_4_C. In the statistical analysis, of all the parameters' influence, high-strength reinforced particles were recorded with strong influence, which was proved in the wear analysis. Hence, the boron carbide particles' influence was placed in the fourth rank.

Increasing the boron carbide percentage from 3% to 6% can cause the minimum wear to occur; further expanding it will lead to an increase in the wear. The highest percentage level (0.8%) of MWCNT offered minimum wear of the magnesium composites, as shown in Figure 6. The minimum period of ball milling produced low wear. Similarly, 3 h of sintering temperature offered minimum wear. The Pareto chart clearly shows the higher and lower effects of the parameters in the wear analysis, as shown in Figure 7. Furthermore, this plot signifies which parameter was statistically significant, indicating the significance by *α* or alpha. Bars in the Pareto charts that crossed the reference lines were statistically significant. Ball milling and MWCNT parameters crossed the reference lines; hence, these parameters are producing essential effects in wear analysis and are statistically significant at the 0.05 level in the selected model.

Table 6 presents the higher contribution levels of the parameters in the wear analysis. The ball milling parameter contributed enormously (60.79%), followed by MWCNTs (15.59%), sintering process (6.69%), and boron carbide reinforcement percentage (1.59%).

The regression equation is as follows:

Wear (*g*) = −0.00614 + 0.000525 B_4_C (%) − 0.02463 MWCNT (%)

Figure 8 represents the contour plot of the wear analysis.  Figure 8(a) shows the influence of two parameters such as B_4_C% and MWCNT. Maximum levels of both the parameters offered minimum wear.  Figure 8(b) illustrates that 0.8% of MWCNTs and 3 h of the ball milling process produced minimum wear.  Figure 8(c) shows that 3 h of ball milling and 4 h of sintering recorded the minimum wear.  Figure 8(d) exemplifies that 9% of MWCNTs and the 5 h sintering process registered the minimum wear.

### 4.2. Microhardness Analysis

The multiwall carbon nanotube percentage parameter highly influenced the microhardness analysis and is presented in the response Table 7 (means) and Table 8 (S/N ratio). Furthermore, B_4_C (%) had a high influence, followed by ball milling and sintering. Optimal parameters were attained at 12% of boron carbide, 0.4% of MWCNT, 4 h of the ball milling process, and 6 h of the sintering process. In microhardness analysis, both reinforced particles such as boron carbide and multiwall carbon nanotubes were blended significantly. It was noticed in the rank order. The ball milling process was used to improve the blending of the particles. It made high-strength composites. These three parameters had a high influence; hence, the influence of the sintering time parameter was less than that of other microhardness analysis parameters. Increasing boron carbide percentage increased the microhardness of the magnesium composites, as shown in Figure 9. A higher rate (12%) of boron carbide offered extreme microhardness. 0.4% of MWCNT and 4 h of ball milling produced higher microhardness values. A higher sintering time (6 h) offered excellent microhardness.

Higher effects of the parameters were illustrated in the Pareto chart, as shown in Figure 10. This plot expresses whether the parameters were statistically significant or not at the optimum level. From the microhardness analysis, three parameters had a high influence: boron carbide percentage, ball milling hours, and MWCNT percentage. These parameters crossed the reference line; hence, these parameters mainly affected the microhardness, and they are statistically significant (*P* value = 0.05).

From Table 9, the higher contribution parameters were identified, such as 24% contribution by boron carbide followed by 19.69% contribution by the ball milling process, 14.95% by MWCNT, and 8.52% by the sintering process. The *P* value of all parameters was less than 0.05. Hence, the parameter's influence was insignificant, and the chosen model was excellent.

The regression equation is as follows:

Microhardness (HV) = 41.6 + 5.38 B_4_C (%) − 62.8 MWCNT (%) + 14.30 ball milling (*h*) + 9.48 sintering (h)

Figure 11 presents the 3D surface plot for microhardness analysis; 0.6% of MWCNTs and 8% of boron carbide correlations offered higher microhardness values, as shown in Figure 11(a).  Figure 11(b) illustrates the links between MWCNT % and ball milling time; 0.4% of MWCNT and 4 h of ball milling provided excellent microhardness.  Figure 11(c) represents the connection between ball milling and sintering process, both the parameters at 4 h period recorded a maximum microhardness value.  Figure 11(d) illustrates the correlation between sintering and B_4_C %; in this analysis, 4 h of sintering time and 12% of boron carbide offered superior microhardness values.

### 4.3. Salt Spray Analysis

Among all four parameters, the sintering process parameter had an exceptional influence in the salt spray corrosion test as presented in the response Table 10 (means) and Table 11 (S/N ratio). Further followed by the parameter were B_4_C %, ball milling process, and MWCNT (%) in the rank order. In the salt spray corrosion test analysis, optimal parameters obtained were 3% boron carbide, 0.4% MWCNT, 4 h of the ball milling process, and 3 h of the sintering process.

A lower level (3%) of boron carbide percentage offered the minimum corrosion rate. Further increasing boron carbide percentage increased the corrosion rate as shown in Figure 12. A moderate level (0.4%) of multiwall carbon nanotube percentage produced a minimum corrosion rate, and continually increasing the percentage of MWCNTs decreased the corrosion rate. Gradually increasing the ball milling process time from 1 h to 4 h recorded a minimum corrosion rate. Increasing the sintering time from 3 h to 6 h increases the corrosion rate; 3 h sintering offers a minimum level of corrosion rate.

Figure 13 presents the higher effects of the parameters in the Pareto chart. From this chart, only the boron carbide percentage crossed the reference line and was denoted as a statistically significant parameter compared to other parameters. The sintering time parameter nearly touches the reference line but has not crossed the mentioned level. The other two parameters were not significant such as MWCNTs and ball milling.

The higher contribution was observed at 21.19% by the influence of boron carbide percentage, followed by sintering time (17.96%), ball milling process (16.38%), and MWCNTs percentage (3.07%).  Table 12 presents the *F*-value and *P* value in a transparent manner, and a higher *F*-value (5.63) was obtained by the influencing boron carbide percentage parameter.

The regression equation is as follows:

Corrosion rate (mm/yr) = −0.00172 + 0.000245 B_4_C (%) + 0.00140 MWCNT (%) − 0.000645 ball milling (h) + 0.000675 sintering (h)

Figure 14 presents the 3D trajectory plot for corrosion rate analysis by correlating the two parameters involved.  Figure 14(a) showed the correlation between B_4_C % and MWCNT %, from that the 12% of boron carbide and 0.4% of MWCNTs recorded the lower level of corrosion rate.  Figure 14(b) represents 0.4% of MWCNTs and 3 h of the ball milling process produced the minimum corrosion rate.  Figure 14(c) illustrates the 3 h ball milling and 3 h sintering time decreased the corrosion rate and offered a minimum corrosion rate.  Figure 14(d) represents that 4 h of sintering time and reinforcement of 6% of boron carbide produces a minimum corrosion rate.

Figure 15 illustrates the wear and corrosion test SEM images. Figures 15(a) and 15(b) demonstrate that the SEM image was taken before the wear test and corrosion test, respectively; it visibly showed the dispersions of B_4_C and MWCNT particles. The corrosion test specimen image identified the deep groove due to improper blending of particles in the P/M process. Figures 15(c) and 15(d) illustrate that the SEM image was taken after the wear and corrosion tests. The photos show defects such as delamination, continuous groove, black regions, and debris. These defects were noticed which shows that some deviations were present in the sintering process.

## 5. Conclusion

Using the powder metallurgy process, the hybrid magnesium composites were prepared with boron carbide and multiwall carbon nanotubes with different percentage levels. The wear, microhardness, and corrosion rates of the composites were examined through the Taguchi statistical tool. Furthermore, the parameters of the P/M process were optimized, and the results were discussed and exhibited as follows:

  From the wear analysis, the minimum wear was 0.007 g with an influence of 9% boron carbide, 0.8% MWCNT, 2 h of the ball milling process, and 3 h of the sintering process. In microhardness analysis, maximum hardness was 181.4 HV by 12% boron carbide, 0.2% of MWCNT, 4 h of the ball milling process, and 4 h of the sintering process. In corrosion rate inspection, the minimum corrosion rate was 0.00078 mm/yr by 12% boron carbide, 0.4% of MWCNT, 3 h of the ball milling process, and 3 h of the sintering process.
  In wear analysis, the optimal parameters were 12% of boron carbide, 0.4% of MWCNT, 4 h of the ball milling process, and 6 h of the sintering process. In microhardness analysis, the optimal parameters were 12% boron carbide, 0.4% MWCNT, 4 h of the ball milling process, and 6 h of the sintering process. Finally, in corrosion rate analysis, the optimal parameters were 3% of boron carbide, 0.4% of MWCNT, 4 h of the ball milling process, and 3 h of the sintering process. The revolutionary blending of reinforced particles and its sintering process moderately improved the hardness value. Similarly, it enhanced the wear and corrosion resistance of the hybrid composites.
  In wear analysis, the ball milling parameter highly contributed at 60.79%. In microhardness analysis, the boron carbide percentage level contributed 24.65%. Similarly, in corrosion rate analysis, boron carbide contributed 21.19%. The high contribution of boron carbide reduced the corrosion rate and increased the microhardness through the homogeneous mixture of the B_4_C and MWCNT into the AZ80.
  From the ball milling mechanism, by increasing the ball-milling time, the powder particles were blended homogeneously, which was reflected in the wear analysis as minimum wear. Using the sintering mechanism, green compact specimens were firmly converted into high-hardness specimens due to melted particles sticking to each other, reducing the corrosion rate. The novelty of adding the MWCNT particles improved the microhardness of the magnesium alloy hybrid composites.

## Figures and Tables

**Figure 1:** Ball milling process.

**Figure 2:** Cold compaction process.

**Figure 3:** Sintering process.

**Figure 4:** Sintered specimens: (a) before sintering; (b) after sintering.

**Figure 5:** Dry sliding wear test apparatus.

**Figure 6:** Main effects plot for wear analysis: (a) means; (b) S/N ratio.

**Figure 7:** Pareto chart for wear analysis.

**Figure 8:** Contour plot for wear analysis: (a) B_4_C % vs. MWCNT; (b) MWCNT vs. ball milling; (c) ball milling vs. sintering; (d) sintering vs. MWCNT.

**Figure 9:** Main effects plot for microhardness analysis: (a) means (b) S/N ratio.

**Figure 10:** Pareto chart for microhardness analysis.

**Figure 11:** 3D Surface plot analysis for microhardness: (a) B_4_C % vs. MWCNT (%); (b) MWCNT (%) vs. ball milling; (c) ball milling vs. sintering; (d) sintering vs. B_4_C %.

**Figure 12:** Main effects plot for corrosion analysis: (a) means (b) S/N ratio.

**Figure 13:** Pareto chart for corrosion rate analysis.

**Figure 14:** 3D trajectory plot for corrosion rate: (a) B_4_C % vs MWCNT (%); (b) MWCNT (%) vs. ball milling; (c) ball milling vs. sintering; (d) sintering vs. B_4_C %.

**Figure 15:** SEM images: (a) before wear test; (b) before corrosion test; (c) after wear test; (d) after corrosion test.

**Table 1:** Chemical composition of AZ80 magnesium alloy.

Element	Contribution (%)
Aluminum (Al)	8.20
Zinc (Zn)	0.60
Manganese (Mn)	0.10
Silicon (Si)	0.12
Copper (Cu)	0.045
Iron (Fe)	0.0040
Nickel (Ni)	0.0050
Magnesium (Mg)	Balance.

**Table 2:** Process parameters and their levels of the P/M process.

Parameters	Level 1	Level 2	Level 3	Level 4
B_4_C (%)	3	6	9	12
MWCNT (%)	0.2	0.4	0.6	0.8
Ball milling (h)	1	2	3	4
Sintering (h)	3	4	5	6

**Table 3:** Experimental summary of the P/M process parameters and the results.

Exp. Runs	B_4_C (%)	MWCNT (%)	Ball milling (h)	Sintering (h)	Wear (g)	Microhardness (HV)	Corrosion rate (mm/yr)
1	3	0.2	1	3	0.008	84.3	0.00085
2	3	0.4	2	4	0.031	120.5	0.00147
3	3	0.6	3	5	0.025	90.6	0.00232
4	3	0.8	4	6	0.037	115.9	0.00128
5	6	0.2	2	5	0.022	87.3	0.00204
6	6	0.4	1	6	0.009	168.6	0.00291
7	6	0.6	4	3	0.034	144.4	0.00097
8	6	0.8	3	4	0.008	99.3	0.00083
9	9	0.2	3	6	0.047	179.8	0.00307
10	9	0.4	4	5	0.041	177.3	0.00119
11	9	0.6	1	4	0.008	92.4	0.00246
12	9	0.8	2	3	0.007	89.3	0.00118
13	12	0.2	4	4	0.044	181.4	0.00282
14	12	0.4	3	3	0.031	165.9	0.00078
15	12	0.6	2	6	0.028	155.3	0.00344
16	12	0.8	1	5	0.009	110.6	0.00827

**Table 4:** Response table for means (wear).

Level	B_4_C (%)	MWCNT (%)	Ball milling (h)	Sintering (h)
1	0.025250	0.030250	0.008500	0.020000
2	0.018250	0.028000	0.022000	0.022750
3	0.025750	0.023750	0.027750	0.024250
4	0.028000	0.015250	0.039000	0.030250
Delta	0.009750	0.015000	0.030500	0.010250
Rank	4	2	1	3

**Table 5:** Response table for signal-to-noise ratios (wear). Smaller is better.

Level	B_4_C (%)	MWCNT (%)	Ball milling (h)	Sintering (h)
1	33.20	32.19	41.43	36.14
2	36.34	32.25	34.37	35.30
3	34.83	33.60	32.68	33.46
4	32.32	38.65	28.22	31.79
Delta	4.02	6.45	13.21	4.35
Rank	4	2	1	3

**Table 6:** Analysis of variance for wear analysis.

Source	DF	Seq SS	Contribution (%)	Adj. SS	Adj. MS	*F*-value	*P* value
Regression	4	0.002634	84.66	0.002634	0.000659	15.18	0.000
B_4_C (%)	1	0.000050	1.59	0.000050	0.000050	1.14	0.308
MWCNT (%)	1	0.000485	15.59	0.000485	0.000485	11.18	0.007
Ball milling (h)	1	0.001892	60.79	0.001892	0.001892	43.60	0.000
Sintering (h)	1	0.000208	6.69	0.000208	0.000208	4.80	0.051
Error	11	0.000477	15.34	0.000477	0.000043		
Total	15	0.003111	100.00				

**Table 7:** Response table for means.

Level	B_4_C (%)	MWCNT (%)	Ball milling (h)	Sintering (h)
1	102.8	133.2	114.0	121.0
2	124.9	158.1	113.1	123.4
3	134.7	120.7	133.9	116.4
4	153.3	103.8	154.7	154.9
Delta	50.5	54.3	41.6	38.5
Rank	2	1	3	4

**Table 8:** Response table for signal-to-noise ratios. Larger is better.

Level	B_4_C (%)	MWCNT (%)	Ball milling (h)	Sintering (h)	
1	40.14	41.90	40.81		41.28
2	41.62	43.88	40.82		41.51
3	42.10	41.37	42.14		40.95
4	43.57	40.28	43.65		43.68
Delta	3.43	3.60	2.84		2.73
Rank	2	1	3		4

**Table 9:** Analysis of variance for microhardness values.

Source	Df	Seq. SS	Contribution (%)	Adj. SS	Adj. MS	*F*-value	*P* value
Regression	4	14246	67.52	14246	3561.5	5.72	0.010
B_4_C (%)	1	5200	24.65	5200	5200.4	8.35	0.015
MWCNT (%)	1	3155	14.95	3155	3155.2	5.06	0.046
Ball milling (h)	1	4092	19.39	4092	4092.2	6.57	0.026
Sintering (h)	1	1798	8.52	1798	1798.1	2.89	0.117
Error	11	6854	32.48	6854	623.1		
Total	15	21100	100.00				

**Table 10:** Response table for means (corrosion).

Level	B_4_C (%)	MWCNT (%)	Ball milling (h)	Sintering (h)
1	0.001480	0.002195	0.003623	0.000945
2	0.001687	0.001590	0.002033	0.001894
3	0.001977	0.002298	0.001749	0.003458
4	0.003828	0.002890	0.001567	0.002675
Delta	0.002348	0.001300	0.002056	0.002513
Rank	2	4	3	1

**Table 11:** Response table for signal-to-noise ratios (corrosion). Smaller is better.

Level	B_4_C (%)	MWCNT (%)	Ball milling (h)	Sintering (h)
1	57.15	54.12	51.49	60.60
2	56.61	56.99	54.57	55.37
3	54.85	53.60	56.69	51.64
4	51.02	54.93	56.88	52.03
Delta	6.14	3.39	5.39	8.96
Rank	2	4	3	1

**Table 12:** Analysis of variance for corrosion rate.

Source	DF	Seq. SS	Contribution (%)	Adj. SS	Adj. MS	*F*-value	*P* value
Regression	4	0.000030	58.60	0.000030	0.000007	3.89	0.033
B_4_C (%)	1	0.000011	21.19	0.000011	0.000011	5.63	0.037
MWCNT (%)	1	0.000002	3.07	0.000002	0.000002	0.82	0.386
Ball milling (h)	1	0.000008	16.38	0.000008	0.000008	4.35	0.061
Sintering (h)	1	0.000009	17.96	0.000009	0.000009	4.77	0.051
Error	11	0.000021	41.40	0.000021	0.000002		
Total	15	0.000051	100.00				

## Data Availability

The data used to support the findings of this study are included in the article. Further data or information are available from the corresponding author upon request.
